# Bachu Mushroom Polysaccharide Alleviates Colonic Injury by Modulating the Gut Microbiota

This article has been retracted.

**DOI:** 10.1155/2022/1353724

**Published:** 2022-03-14

**Authors:** Zumrat Abdureyim, Lei Wang, Qing Tao, Jing Xu, Delixiati Yimiti, Qian Gao

**Affiliations:** ^1^Department of Labor Hygiene and Environmental Hygiene, College of Public Health, Xinjiang Medical University, Urumqi, 830017 Xinjiang, China; ^2^Key Laboratories of Molecular Medicine of Jiangsu Province, Nanjing University School of Medicine, Nanjing, 210003 Jiangsu, China; ^3^Department of Clinical Laboratory, Jiangsu Province Hospital on Integration of Chinese and Western Medicine, Jiangsu Province Academy of Traditional Chinese Medicine, Nanjing 210028, China

## Abstract

**Objective:**

This study was to define the protective effect of purified *Helvella leucopus* polysaccharide (p-HLP) against dextran sulfate sodium- (DSS-) induced colitis.

**Methods:**

The novel p-HLP was isolated from Bachu mushroom through hot water extraction, ethanol precipitation, and column chromatography. Then, we evaluated the potential effects of p-HLP on colonic histopathology, inflammation, and microbiota composition in DSS-induced colitis mice.

**Results:**

p-HLP was a homopolysaccharide with an average molecular weight of 39.14 × 10^8^ Da. Functionally, p-HLP significantly attenuated DSS-induced body weight loss and colon shortening. The histological score of the colon lesion was significantly decreased upon p-HLP treatment. Also, p-HLP treatment led to decreased expression of proinflammatory cytokines and mediators (IL-6, IL-1*β* and TNF-*α*, and COX-2 and iNOS) and increased expression of anti-inflammatory cytokine (IL-10) in the colon tissues. Illumina MiSeq sequencing revealed that p-HLP modulated the composition of the gut microbiota.

**Conclusion:**

p-HLP is a potent regulator that protects the lesions from DSS-induced colitis.

## 1. Introduction

Inflammatory bowel disease (IBD), an umbrella term for chronic and recurrent inflammation in the digestive tract, is characterized by abdominal pain, chronic diarrhea, rectal bleeding fatigue, and weight loss [1]. IBD encompasses ulcerative colitis and Crohn's disease, and this disease has become a noticeable public health burden worldwide with increasing prevalence [2]. Although the precise pathogenic mechanism of IBD is not fully understood, a complex interaction between IBD-related etiologies, including host genetics, environmental risk factors, immune dysfunction, and dysregulation of the gut microbiota, has been associated with the risk of IBD onset and progression [3].

Unbalanced expression of cytokines, such as increased production of proinflammatory cytokines IL-6, IL-1*β*, and TNF-*α* and decreased production of anti-inflammatory cytokine IL-10 and IL-4, is coupled to the risk of acute colitis [4]. Such an abnormal expression leads to mucosal injury and consequent epithelial barrier damage, aberrant immune responses, and dysbiosis of gut microbiota associated with functional changes in the microbial metabolome [5]. The changes of gut microbiota may in turn affect the physiology and immunology of the host [6–8].

Previously, various treatments including aminosalicylate, corticosteroids, immunomodulators, Janus kinase inhibitors, and biological therapies [9–11] have been evidenced as beneficial to IBD; however, these drugs may also have limitations, which are mainly the high recurrences of clinical manifestations, long treatment cycles, and low responses to initial treatment [12]. Therefore, it is desirable to identify healthy and natural compounds with IBD prevention activity. Latterly, novel therapeutic options based on gut microbiota modulation have been suggested [13]. For examples, the *in vitro* and *in vivo* anti-inflammatory effects of several natural compounds, including the edible mushroom polysaccharides (MPs), have been critically studied for their nontoxicity and high efficiency [14, 15]. The administrations of MPs, as shown in various clinical studies, contribute to the integrity of intestinal mucosa by regulating inflammatory responses and the gut microbiota in IBD patients [16].

*Helvella leucopus* is distributed in *Populus euphratica* forests in Tarim Basin, also called Bachu mushroom by local residents in Bachu County (Xinjiang, China). Bachu mushroom is an edible and medicinal wild fungus enriched with various bioactive components including polysaccharides, adenosine, cordycepic acid, and minerals [17]. Traditionally, it is broadly used for tuberculosis, fester, bellyache, stomach ailments, hypercholesterolemia, diabetes, and cerebral and cardiovascular diseases [18]. However, so far, no report has connected *Helvella leucopus* polysaccharide (HLP) to the anti-inflammatory effect and the regulation of gut microbial ecosystem in colitis.

## 2. Materials and Methods

### 2.1. Materials and Chemicals

Dried fruit bodies of the Bachu mushroom were obtained from Bachu County in Xinjiang Province, China. All chemical reagents used in high-performance liquid chromatography (HPLC) and ultra-high performance liquid chromatography-tandem mass spectrometry (UPLC-MS/MS) analysis were of mass spectrometry grade and purchased from Thermo Fisher Scientific Inc. (Waltham, MA, USA). Dextran sulfate sodium salt (36–50 kDa) was obtained from MP Biomedicals (Santa Ana, CA, USA). Antibodies against TNF-*α*, IL-6, IL-1*β*, IL-10, iNOS, COX-2, and GAPDH were purchased from KeyGEN Biotech (Nanjing, China).

### 2.2. Extraction and Purification of Polysaccharides from Bachu Mushroom

The dried fruiting bodies of Bachu mushroom were mixed with double-distilled water in the ratio of 1 : 30 (*w*/*v*) and then boiled for 2 h twice. The collected supernatant was combined and concentrated to 1/4 volume at 60°C by a rotary evaporator (RE-2000A, Yarong Co. Ltd., Shanghai, China). After that, the protein content was removed more than 3 times with chloroform : butanol (4 : 1, *v*/*v*) following the Sevag method [19]. The obtained solution was precipitated with 4 volumes of 80% ethanol for 24 h at 4°C. After centrifugation at 12000 r/min for 10 min, the polysaccharides were collected and lyophilized. The residue was dissolved in distilled water (50 mg/mL) and dialyzed with a cellulose membrane (5 kDa) with distilled water at room temperature for 48 h, followed by lyophilization to obtain crude HLP.

The dried aqueous polysaccharide sample (100 mg) was separated by its polarity, was weighed, dissolved in 3 mL of distilled water, and centrifuged at 12000 rpm for 10 min. The supernatant was subjected to purification by using a polysaccharide gel purification system combined with a differential detector (RI-502, Shodex, Tokyo, Japan) for online detection and collection. A symmetrical peak with high polysaccharide content was collected; then, the sample was concentrated by a rotary evaporator at 60°C and lyophilized to obtain purified HLP (p-HLP).

### 2.3. Structural Characterization

#### 2.3.1. Determination of Molecular Weight

The molecular weight of purified HLP was estimated by gel permeation chromatography-refractive index-multiangle laser light scattering (GPC-RI-MALS) (DAWN HELEOS II, Wyatt Technology, Santa Barbara, CA, USA) with slight modification [20]. The eluent was monitored with a refractive index detector (Agilent 1260, USA) coupled with an analytic column (Ohpak SB-805 HQ, Ohpak SB-804 HQ, or Ohpak SB-803 HQ (Shodex, Asahipak, Tokyo, Japan)) for the appropriate molecular weight range. The sample injection volume was 100 *μ*L.

#### 2.3.2. Determination of Monosaccharide Composition

After dialysis and lyophilization, the monosaccharide composition was analyzed by a Thermo ICS5000+ chromatography system (Thermo Fisher Scientific, MMAS, USA) with a Dionex™ CarboPac™ PA200 column as described previously with some modifications [20].

#### 2.3.3. Determination of Glycosidic Linkages

Reduction of uronic acid was performed according to the protocol reported by Taylor and Conrad [21]. Then, the obtained reduced substances were subjected to methylation analysis as described by Anumula and Taylor [22] with some modifications. In this procedure, 10 mg of polysaccharide was dissolved in DMSO/NaOH and incubated for 30 min. After incubation, methyl iodide solution was added for 1 h reaction, and then, the samples were methylated with CH3I. The methylated products were hydrolyzed with trifluoroacetic acid (TFA, 2 mol/L, 100 *μ*L) at 121°C for 90 min. After reduction, the hydrolysates were converted to partially methylated alditol acetates (PMAAs) and analyzed by electron ionization mass spectrometry (EI-MS, Agilent 7890A/5977B, USA).

### 2.4. Animals and Experimental Design

Male C57BL/6 mice (SPF grade, 6–8 weeks old) were purchased from the Model Animal Research Center of Nanjing University, and five mice were housed per cage under a 12–12 h light/dark cycle at 20–22°C and 55 ± 5% relative humidity for one week before the experiment. For each group of experiments, mice were matched by body weight. All experimental procedures and protocols were approved by the Institutional Animal Care and Use Committee of Nanjing University, Nanjing, China (Approval No. JN. No2018-035210-225A).

After adaption, experimental subjects were randomly assigned to 5 groups (*n* = 5 each group): the negative control (NC) group, dextran sulfate sodium (DSS) model group, p-HLP group, low-dose p-HLP (DSS+p-HLP(L)) group, high-dose p-HLP (DSS+p-HLP(H)) group, and p-HLP group. NC group mice received drinking water from day 0 to day 7. DSS group mice were allowed access to water containing 3% DSS for 7days to induce ulcerative colitis, and water was replaced every other day. In the DSS+p-HLP(L) group, mice were treated by oral gavage with p-HLP (10 mg/kg BW/d) for 7days combined with DSS induction same as the DSS group. In the DSS+p-HLP(H) group, mice were orally administered with p-HLP (50 mg/kg BW/d) for 7 days combined with DSS induction same as the DSS group. In the p-HLP group, mice received normal drinking water and orally administered with p-HLP (100 mg/kg BW/d) for 7days. As shown in Table S1, the disease activity index (DAI) was recorded daily, which is the combined score of body weight loss, stool consistency, and bleeding [23]. On day 8, all animals were sacrificed to collect colon tissue, spleen, and fecal samples. Then, the colon length and spleen weight were measured.

### 2.5. Histopathological Analysis

The colon samples were rinsed with cold PBS (phosphate-buffered saline), and then, the distal part of each colon was fixed with 10% paraformaldehyde and embedded in paraffin. Tissue sections (5 *μ*m) were stained with hematoxylin-eosin (HE) for histological evaluation and microscopic analysis. The histological score was also evaluated based on a previously described method [24] for DSS-induced colitis (Table S2).

### 2.6. RNA Isolation and RT-qPCR

Total RNA was isolated from the colonic tissues using the FastPure Cell/Tissue Total RNA Isolation Kit (Vazyme, Nanjing, Jiangsu, China), and cDNA was obtained using the PrimeScript™ RT Master Mix (TaKaRa, Beijing, China). Real-time quantitative polymerase chain reaction (RT-qPCR) was conducted in triplicate on a QuantStudio 5 (Thermo Fisher Scientific, Shanghai, China) using the PowerUp™ SYBR™ Green Master Mix (Thermo Fisher Scientific, Shanghai, China) according to the manufacturer's protocol. The relative amount of each transcript was normalized to the expression of the housekeeping gene (GAPDH), and data were analyzed according to the 2^-*ΔΔ*Ct^ method. The primer sequences for TNF-*α*, IL-1*β*, IL-6, IL-10, iNOS, and COX-2 are shown in Table S3.

### 2.7. DNA Extraction and PCR Amplification

Microbial DNA was extracted from colonic samples using the E.Z.N.A.® Soil DNA Kit (Omega Bio-Tek, Norcross, GA, U.S.). The V4 region of the bacterial 16S rRNA gene was amplified using the primers 515F (5′-barcode-GTGCCAGCMGCCGCGG-3′) and 806R (5′-GGACTACNVGGGTWTCTAA-3′). The PCR products were examined by 2% agarose electrophoresis, purified using the AxyPrep DNA Gel Extraction Kit (Axygen Biosciences, Union City, CA, U.S.), and quantified by Qubit®3.0 (Life Invitrogen) according to the manufacturer's instructions. The amplicons were normalized, pooled, and paired-end sequenced (2 × 250) on an Illumina MiSeq platform (Shanghai Biozeron Co., Ltd.). Merged reads were analyzed with QIIME v2, and low-quality reads were removed. After paired read merging and chimera filtering, the phylogenetic affiliation of each 16S rRNA gene sequence (herein, called RSVs) was analyzed by the RDP Classifier (http://rdp.cme.msu.edu/) against the SILVA (SSU132) 16S rRNA database using a confidence threshold of 70%. Finally, operational taxonomic units (OTUs) were classified using BLASTn against a curated database derived from Greengenes, RDPII, and NCBI. LEfSe (linear discriminant analysis (LDA) effect size) analysis was performed to determine the size effect of each distinctively abundant taxon [25]. A significance value of <0.05 combined with an effect size threshold of 4 was used for LEfSe analysis.

### 2.8. Statistical Analysis

Statistical analysis was performed by using two-way analysis of variance (ANOVA) or one-way ANOVA followed by Tukey's multiple comparison with SPSS 22.0 software (IBM, Chicago, IL, USA). Data are presented as the mean ± standard deviation (SD) or as box-and-whisker plots unless otherwise indicated, and *P* < 0.05 was considered statistically significant.

## 3. Results

### 3.1. Characterization of Compositional Features of p-HLP

The crude p-HLP was initially isolated by water extraction along with alcohol precipitation with approximately 4.25% of original weight of the dry powder of Bachu mushroom. After isolation, the highest yielding independent elution peak fraction was further purified by a polysaccharide gel purification system combined with a differential detector. A single, symmetrical, and narrow peak that indicated as a homogeneous polysaccharide was eluted (Figure 1(a)). The fraction was collected, concentrated, and lyophilized with a yield of approximately 2.8% of crude polysaccharides in weight, and it was designated as p-HLP.

Next, the molecular weight, the monosaccharide composition, and the nature of glycosidic linkage of p-HLP were characterized using GPC-RI-MALS, ion chromatography (IC), and gas chromatography-mass spectrometer (GC–MS), respectively. As shown in Table 1 and Figure 1(b), we yielded an average molecular weight (Mw) of 39.14 × 10^8^ Da, a *z*-average molecular weight (Mz) of 18.95 × 10^8^ Da, a number average molecular weight (Mn) of 93.84 × 10^8^ Da, and a polydispersity (Mw/Mn) of 2.07.

The monosaccharide composition of p-HLP was determined, which mainly contained mannose (43.68%), glucose (38.16%), rhamnose (9.34%), and galactose (4.35%); the above four accounted for more than 95% (95.53%) of the total monosaccharide in p-HLP. The monosaccharides also included low levels of fucose (0.88%), xylose (0.84%), GalA (0.79%), Glc-UA (0.74%), Gul-UA (0.72%), and arabinose (0.50%) (Figure 1(c), Table 1). In addition, a total of eleven different linked residues were identified, with four nonreducing termini that are glucose (T-D-Glc, 8.48%), rhamnose (T-D-Rha, 6.05%), mannose (T-D-Man, 5.50%), and galactose (T-D-Gal, 0.70%), as well as seven nonterminal saccharide residues that are 4-Glc*p*, 2-Man*p*, 6-Man*p*, 3,6-Man*p*, 4,6-Gal*p*, 6-Glc*p*, and 3-Glc*p* with molar ratios of 31.60 : 28.71 : 8.22 : 4.29 : 2.74 : 2.15 : 1.58, respectively (Table S4).

### 3.2. p-HLP Potently Attenuated DSS-Induced Acute Colitis Symptoms

Next, the function of p-HLP was tested in a colitis mouse model (3% DSS, Methods). As presented in Figure 2, DSS treatment caused a significant body weight loss (Figures 2(a) and 2(b)), whereas the administration of p-HLP, especially at a high dose (50 mg/kg), significantly reversed the body weight loss (*P* <0.01) (Figures 2(a) and 2(b)). Both low and high doses of p-HLP markedly alleviated the DAI compared with that of the DSS group (Figure 2(c)). Also, the DSS-induced colon shortening was significantly suppressed by both low and high doses of p-HLP (*P* < 0.05 and *P* < 0.01, respectively) (Figures 2(d) and 2(e)). Moreover, DSS induced a significant increase in the spleen index (the ratio of spleen weight to body weight), whereas the index returned to near normal levels in both low and high p-HLP-dosed animals (*P* < 0.01) (Figure 2(f)). No significant difference, it should be noted, was identified between the NC group and the p-HLP alone group in all the tests, suggesting that p-HLP at the tested level (100 mg/kg BW/d) had no detectable effect on mice.

### 3.3. DSS-Induced Gut Lesions Were Ameliorated with p-HLP Treatment

We further investigated the therapeutic value of p-HLP in DSS-induced colitis by HE staining. As shown in Figures 3(a) and 3(e), the NC group and the p-HLP alone group showed normal morphology of the colons, including a complete mucosal layer accompanied by well-arranged crypts, rich intestinal glands, and goblet cells. In contrast, the administration of DSS induced the severe damage on the colon epithelium, the pronounced decrease in the number of crypts, and the infiltration of inflammatory cells in the muscular layer in the colon tissues (Figure 3(b)). However, p-HLP treatment, especially at a high dose, relieved the histological lesions, resulting in a relatively intact epithelium and glandular structure and causing regenerative crypts, along with less inflammatory cell infiltration and mild submucosal edema (Figures 3(c) and 3(d)). The histological index in the DSS-induced mice was markedly reduced after the high dose of p-HLP (*P* < 0.001) (Figure 3(f)), although the low dose of p-HLP showed a reduced protective effect in the histological index (Figure 3(f)).

### 3.4. p-HLP Reduced the Expression of Inflammatory Genes in Colitis Colon

We next measured the mRNA levels of inflammatory cytokines and factors (IL-6, IL-1*β*, TNF-*α*, IL-10, iNOS, COX-2) in the colon tissues by RT-qPCR. As expected, DSS treatment resulted in increases in the levels of proinflammatory cytokine IL-6, IL-1*β*, and TNF-*α* and proinflammatory factors iNOS and COX-2 (*P* < 0.01) (Figures 4(a)–4(f)) and decreases in the anti-inflammatory cytokine IL-10 (*P* < 0.01) (Figure 4(d)). p-HLP administration, specifically at a high dose, markedly downregulated the productions of IL-6, IL-1*β*, TNF-*α*, and iNOS and COX-2, and upregulated IL-10, when compared with those of the DSS group (*P* < 0.01) (Figures 4(a)–4(f)). The mRNA levels of inflammatory cytokines and factors were not changed in the p-HLP alone group when compared to those in the NC group (Figures 4(a)–4(f)).

### 3.5. p-HLP Regulated the Gut Dysbiosis in DSS-Induced Colitis

To assess the effect of p-HLP on gut microbiota, we conducted a 16S rRNA sequencing analysis with a high sequencing depth. The rarefaction curves of all tested groups have reached their plateaus, indicating that the sequencing depth was adequate (Figure S1A). The alpha diversities presented as *Shannon*, *Chao1*, and *Simpson* indices were used to estimate the richness/evennes*s* of the gut microbiota in each group. Compared with normal mice, the *Shannon* and *Chao1* indices exhibited a reduction after a high dose of p-HLP treatment (Table S5). A Venn diagram revealed the shared and unique operational taxonomic units (OTUs) across the groups (Figure S1B). A total of 1632 OTUs were shared by all the groups. Notably, the unique numbers of OTUs in the NC and p-HLP(H) groups were slightly reduced (from 853 to 823), while the changes of the unique detected OTUs in DSS (730) vs. p-HLP(L) (812) and p-HLP(H) (569) were bidirectional. Nevertheless, the high-dose P-HLP treatment reduced the number of unique gut OTUs in both NC and DSS backgrounds (*P* < 0.05).

The compositions of the gut microbiota at the phylum and genus levels were assessed and presented in stacked histograms (Figure S1C, D). The top five phyla were actually shared in all groups and were *Firmicutes*, *Bacteroidetes*, *Proteobacteria*, *Verrumicrobiota*, and *Epsilonbacteraeota*, accounting for >98% of the total microbes (Figure S1C, Table 2). In the NC group, the proportion of *Firmicutes* was greater than that of *Bacteroidetes*, whereas in the DSS group, the relative abundances of the two were more alike each other (*P* < 0.05) (Figure S1C). However, the trends of the changes of *Firmicutes* and *Bacteroidetes* abundances in low and high p-HLP-dosed groups were different. In the low-dose p-HLP group, the abundances of the two phyla were as those in the NC group (Figure S1C), while in the high-dose p-HLP-treated mice, *Bacteroidetes* was significantly higher than *Firmicutes* (*P* < 0.05) (Figure S1C). Interestingly, compared with the other four groups, the relative abundances of *Verrumicrobiota* and *Proteobacteria* in the p-HLP alone group were significantly increased and accounted for approximately 30% of the total OTUs (*P* < 0.01) (Figure S1C).

The compositions of the gut microbiota were also analyzed at the genus levels. The genera with relative abundance less than 0.1% were not analyzed. Eventually, 20 genera constituting >78% of the total gut microbiota were selected for analysis (Figure S1D; Table 3). The results showed the genera *Muribaculaceae_norank* occupied an obvious leading role in the microbiota composition of the DSS mice with/without p-HLP treatment, while two *Lachnospiraceae* genera, *Lachonospiraceae_NK4A136_group* and *Lachnospiraceae_unclassified*, were increased in DSS animals but reducing along with p-HLP treatment in a dose-sensitive manner (Figure 5(a)). In contrast, there was an increase in the relative abundance of *Lactobacillus* in the p-HLP(L) and p-HLP(H) groups compared with that in the DSS group (Figure 5(a)).

The beta diversity described the structural variability of the gut microbiota as whole between the groups. With the NC group positioned at the central-basal area in the space defined by PC1 (33.26%) and PC2 (23.63%), the DSS group was on the top of the NC group, while the p-HLP, p-HLP(L), and p-HLP(H) groups were distributed either left or right to the NC group (Figure 5(b)), indicating that the main differences of the microbes between DSS and NC as well as p-HLP-treated mice were in the PCA2.

LEfSe analysis further determined the microorganisms with significant differences among the five groups at different taxonomic levels (Figures 5(c) and 5(d)). Overall, we observed a general enrichment of the family Lactobacillaceae in NC group, while Lachnospiraceae was enriched in the DSS group. Moreover, the high dose of p-HLP increased the abundance of Bacteroidaceae and Prevotellaceae, and Akkermansiaceae was the most distinct taxa at the family level of the p-HLP alone group.

To estimate the overall function of gut microbiotas that was altered after DSS and p-HLP treatment, we employed the Tax4Fun2 analysis, an R package for the prediction of habitat-specific functional profiles and functional redundancy based on 16S rRNA gene sequences. The NC, DSS, and p-HLP(H) groups were selected in this section since they had the most distinct phenotypical characteristics. According to analysis, the pathway of amoebiasis was significant in abundance of the three groups (https://www.genome.jp/kegg-bin/show_pathway?ko05146), with a high level of the readout in the NC group and a significant reduction in the DSS group; the reduction was reversed in the p-HLP(H) group (Figure 5(d)). The results suggested an increased suppression of inflammatory responses, and a potential immunosuppression in NC and p-HLP animals. Such results were consistent with the findings in Section 3.4 regarding inflammatory cytokines and factors. More studies on rigorous data are warranted to further dissect the complex mechanism of p-HLP function on dysbiosis in colitis.

## 4. Discussion

Accumulating evidences have demonstrated that MPs posed favorable therapeutic and health-promoting properties, including anticancer [26], antiviral [27], anti-inflammatory effects [28], and immunomodulatory function [29]. Bachu mushroom is an edible and medicinal mushroom and traditionally used for the treatment of various diseases including digestive diseases, such as stomach ailments [18]. However, Bachu mushroom, especially p-HLP, has not been studied in colitis.

In this paper, the polysaccharide from the Bachu mushroom was purified followed by determination of structure features of p-HLP, and the effect of p-HLP in DSS-induced colitis was studied. The p-HLP with the Mw of 93.84 × 10^8^ Da was identified, which is different from two previously defined Bachu mushroom polysaccharides, HLP1-1 and HLP2-1, with the Mw of 21,382 Da and 23,038 Da, respectively [30]. Meanwhile, the main compositions of the monosaccharides and their molar ratios in p-HLP were different from those in HLP1-1 and HLP2-1. The main monosaccharide composition of p-HLP included mannose, glucose, rhamnose, and galactose with molar ratios of 43.68 : 38.16 : 9.34 : 4.35, while HLP1-1 including mannose, rhamnose, and glucosamine with molar ratios of 78.60 : 11.80 : 1.00 and HLP2-1 including mannose, rhamnose, glucose, and glucosamine with molar ratios of 27.33 : 18.12 : 4.22 : 1.00 [30]. Methylation analysis showed that a total of eleven different linked residues, namely, T-D-Rha, T-D-Man, T-D-Glc, T-D-Gal, 4-Glcp, 2-Manp, 6-Manp, 3,6-Manp, 4,6-Galp, 6-Glcp, and 3-Glcp with molar ratios of 6.05 : 5.50 : 8.48 : 0.70 : 31.60 : 28.71 : 8.22 : 4.29 : 2.74 : 2.15 : 1.58, respectively.

Functional assays showed that after p-HLP treatment, mice with DSS-induced colitis had significant improvement in the DAI score, a comprehensive evaluation metric of disease severity based on weight loss, stool consistency, and occult blood. Furthermore, colon length and spleen index, the additional key indicators reflecting the severity of intestinal inflammation, were also markedly ameliorated upon p-HLP treatment. The histological analysis revealed that p-HLP, particularly at a high dosage, reduced the DSS-induced histological score for measuring pathological symptoms. These results argue that p-HLP treatment effectively protects against DSS-induced colitis.

It has been reported that proinflammatory cytokines play a vital role in intestinal inflammation in IBD [31]. Other proinflammatory factors, such as COX-2 and iNOS, have also been shown to affect the integrity of the colonic mucosa and induce intestinal damage in colitis [32]. However, polysaccharides, especially those isolated from mushrooms, e.g., L-theanine [33], can limit the gut inflammation by reducing the proinflammatory cytokines/mediators and increasing anti-inflammatory cytokines in the colon tissue in colitis [34]. Similarly, we found a potent effect of p-HLP in relieving DSS-induced inflammation in colon tissue in a dose-dependent manner.

The DSS-induced dysregulation of the gut mucosal immune system is believed to introduce excessive immunological responses towards bacteria, leading to alterations in gut microbial composition [35]. As reported, natural polysaccharides can deliver the health benefit potentially through the regulation of the gut microbiota [36]. Therefore, we performed a high-throughput sequencing of the V4 region of bacterial 16S rRNA using an Illumina MiSeq platform, aiming to investigate the impact of p-HLP on the gut microbiota in DSS-induced colitis mice. The beta diversity by the PCA plot suggested that colonic microbial community at the OTU level was significantly changed in DSS mice upon p-HLP treatment. DSS, it should be noted, significantly increased the Lachonospiraceae_NK4A136_group and Lachnospiraceae_unclassified, which is in line with the report that Lachnospiraceae exhibited higher relative abundance in IBD patients and mouse models with more severe colitis [37]. Previous *in vitro* and *in vivo* studies have indicate that consumption of polysaccharides from plants or fungi can effectively alleviate the symptoms of IBD by promoting the growth of beneficial bacteria (i.e., *Akkermansia*, *Bifidobacterium*, and *Lactobacillus*) [38–41]. It is interesting to note that p-HLP also increased the abundance of beneficial bacteria *Lactobacillus*. In addition, p-HLP in normal controls greatly enhanced the abundance of *Akkermansia*, but not in DSS mice. It was also observed that a high dose of p-HLP treatment remarkably increased the population of *Bacteroidetes*, the best carbohydrate-degrading bacteria in the colon, which is consistent with findings in African children consuming high-plant polysaccharide diets [42]. Finally, the result of the prediction of habitat-specific functional profiles suggested an increased suppression of inflammatory responses upon p-HLP treatment, which is consistent with the findings in the section regarding inflammatory cytokines.

## 5. Conclusion

In conclusion, the purified Bachu mushroom polysaccharide has a protective effect on DSS-induced colitis in mice. Such an effect is achieved by its anti-inflammatory activity; specifically, p-HLP can downregulate proinflammatory cytokines (IL-6, IL-1*β*, and TNF-*α*) and proinflammatory mediators (COX-2 and iNOS) and upregulate proinflammatory cytokines(IL-10) in a dose-dependent manner. Additionally, the structure and composition of gut microbiota are altered after p-HLP treatment in mice with DSS-induced colitis; p-HLP significantly promotes *Lactobacillus* and downregulates the abundance of Lachnospiraceae_NK4A136 and Lachnospiraceae_unclassified. Collectively, p-HLP may have the potential to serve as an effective candidate in the treatment of IBD.

## Figures and Tables

**Figure 1:** (a) The fraction purified by DEAE-Sepharose fast flow column. (b) The variation tendencies of molar mass, laser scattering (LS), and refractive index (RI) of APS. The red line shows the varying tendency of the LS of p-HLP with the retention time, and the blue line represents the trend of the RI of p-HLP. The shapes of the red and blue curves indicate the sizes of the polysaccharide molecules and their relative proportions in the tested samples. The black line is the varying tendency of the molar mass of the polysaccharides as a function of the retention time. (c) The ion chromatograms of standard monosaccharides. 1: fucose; 2: rhamnose; 3: arabinose; 4: galactose; 5: glucose; 6: xylose; 7: fructose; 8: ribose; 9: galacturonic acid; 10: glucuronic acid; 11: guluronic acid; ^∗^solvent peak. (d) The ion chromatograms of p-HLP.

**Figure 2:** p-HLP alleviates the clinical symptoms of DSS-induced colitis. Mice were administered 3% DSS in drinking water for 7 days with or without p-HLP (10 g/kg BW/d (low dose) or 50 g/kg BW/d (high dose)). NC: drinking water ad libitum; DSS: 3% (*w*/*v*) DSS drinking water ad libitum; DSS+p-HLP(L): 3% (*w*/*v*) DSS drinking water ad libitum and 10 mg p-HLP/kg BW/d by gavage; DSS+p-HLP(H): 3% (*w*/*v*) DSS drinking water ad libitum and 50 mg p-HLP/kg BW/d by gavage; p-HLP: drinking water ad libitum and 100 mg p-HLP/kg BW/d by gavage. (a) Body weight. (b) Body weight change (%). (c) DSS-induced colonic chronic inflammation as scored by the disease activity index (DAI). (d) Representative images of colon samples. (e) Colon length of mice (cm). (f) The spleen index. Bars represent the mean ± SD (*n* = 5). ^##^*P* < 0.01 vs. NC group. ^∗^*P* < 0.05 and ^∗∗^*P* < 0.01 vs. DSS group.

**Figure 3:** Effects of p-HLP on histological structure of colon tissue in colonic mice after DSS exposure as determined via HE staining. Scale bar = 200 *μ*m. (a) NC group. (b) DSS group. (c) DSS+p-HLP(L). (d) DSS+p-HLP(H). (e) p-HLP group. (f) Histological scores of each group were determined. Black arrow indicates the colonic ulcer and desmoplasia; black arrow indicates the severe damage on muscular layer in the colon tissues by inflammation; red arrow indicates the inflammatory cell infiltration; yellow arrow indicates the edema; blue arrow indicates the regenerative crypts. Bars represent the mean ± SD (*n* = 5). ^###^*P* < 0.001 vs. NC group. ^∗∗^*P* < 0.01 and ^∗∗∗^*P* < 0.001 vs. DSS group.

**Figure 4:** The mRNA expression levels of IL-6 (a), IL-1*β* (b), TNF-*α* (c), IL-10 (d), iNOS (e), and COX-2 (f) in the colon tissue were analyzed by RT-qPCR. Data are presented as the mean ± SD (*n* = 5). ^#^*P* < 0.05 and ^##^*P* < 0.01 vs. NC group.^∗∗^*P* < 0.01 vs. DSS group. ns: not significant.

**Figure 5:** Effect of p-HLP on gut microbiota diversity indices in DSS-induced colitis mice. Letters A–E represent NC, DSS, DSS+p-HLP(L), DSS+p-HLP(H), and p-HLP groups, respectively. (a) Relative abundances of the 3 most typical gut bacteria at the genus level. One-way ANOVA followed by Tukey's test was used to evaluate the statistical significance. The different letters (a and b) represent significant differences between different groups (*P* < 0.05). (b) Beta diversity was measured using PCA plots. Each point represents an individual sample, and the points with different colors belong to different treatments. The distance between pairs of points represent the similarity or difference in the microbial community structures. (c) Cladogram illustrating highly abundant taxa across various treatments. (d) Linear discriminant analysis (LDA) indicates the most differentially abundant bacterial taxa in specific samples.

**Table 1:** Monosaccharide compositions (%), molecular weight, and polydispersity of p-HLP.

Item	Value
Monosaccharide compositions	Ratio (%)
Mannose	43.68
Glucose	38.16
Rhamnose	9.34
Galactose	4.35
Fucose	0.88
Xylose	0.84
Galacturonic acid	0.79
Glucuronic acid	0.74
Guluronic acid	0.72
Arabinose	0.50

Molecular weight	Molar mass (g/mol)
Mw	39.14 × 10^8^
Mz	18.95 × 10^8^
Mn	93.84 × 10^8^

Polydispersity	
Mw/Mn	2.07
Mz/Mn	4.95

Radius mean square (R.M.S.) (nm)	
Rn	17.9
Rw	19.5
Rz	25

Note: p-HLP: purified *Helvella leucopus* polysaccharide; Mw: average molecular weight; Mz: *z*-average molecular weight; Mn: number average molecular weight.

**Table 2:** Relative abundance (%) of mouse cecal microbiota at phylum level.

Index	A	B	C	D	E
Firmicutes	70.96 ± 2.83^a^	45.26 ± 7.36^bc^	49.61 ± 8.81^b^	30.14 ± 13.82^c^	36.94 ± 15.17^bc^
Bacteroidetes	24.56 ± 3.78^a^	48.50 ± 3.92^b^	45.02 ± 11.00^b^	61.10 ± 11.04^c^	28.38 ± 3.89^ad^
Epsilonbacteraeota	0.12 ± 0.12^a^	2.32 ± 3.17^ab^	1.71 ± 1.36^ab^	5.61 ± 3.85^b^	3.59 ± 4.78^ab^
Proteobacteria	3.22 ± 1.44^a^	2.11 ± 1.31^a^	2.39 ± 1.42^a^	1.7787 ± 0.59^a^	15.17 ± 11.40^b^
Verrucomicrobia	0.03 ± 0.03^a^	0.03 ± 0.02^a^	0.31 ± 0.28^a^	0.10 ± 0.06^a^	14.83 ± 6.20^b^
Actinobacteria	0.26 ± 0.08^ab^	0.16 ± 0.08^a^	0.25 ± 0.17^ab^	0.34 ± 0.12^b^	0.29 ± 0.16^ab^
Tenericutes	0.39 ± 0.09	0.44 ± 0.48	0.37 ± 0.33	0.09 ± 0.12	0.43 ± 0.69

A: NC group; B: 3% DSS treatment group; C: 3%DSS+p-HLP(L) group; D: 3%DSS+p-HLP(H) group; E: control+p-HLP group. There is significant difference (*P* < 0.05) if the data are labeled with different letters (a–d) in the same line.

**Table 3:** Relative abundance (%) of top taxa at the genus level.

Genus	A	B	C	D	E
Muribaculaceae_norank	21.35 ± 3.00	34.18 ± 9.41	29.88 ± 10.43	29.51 ± 18.62	23.93 ± 2.28
Lactobacillus	23.48 ± 3.61^a^	3.42 ± 4.36^b^	2.13 ± 2.57^b^	5.76 ± 6.86^b^	19.23 ± 8.59^a^
Lachnospiraceae NK4A136	9.02 ± 4.35^ab^	15.62 ± 3.18^a^	10.00 ± 4.30^ac^	2.38 ± 2.96^b^	5.48 ± 6.86^bc^
Dubosiella	14.01 ± 7.85^a^	6.51 ± 8.78^ab^	5.69 ± 3.45^ab^	4.15 ± 1.19^b^	1.48 ± 1.80^b^
Bacteroides	0.12 ± 0.07^a^	3.22 ± 2.51^a^	3.96 ± 3.90^a^	24.49 ± 24.21^b^	2.63 ± 2.86^a^
Akkermansia	0.03 ± 0.03^a^	0.03 ± 0.03^a^	0.31 ± 0.28^a^	0.10 ± 0.06^a^	14.83 ± 6.00^b^
Ileibacterium	3.20 ± 1.46^a^	1.38 ± 2.24^b^	7.95 ± 1.98^c^	0.72 ± 0.45^b^	0.70 ± 1.01^b^
Alloprevotella	2.20 ± 1.03	5.07 ± 6.01	5.88 ± 8.80	0.08 ± 0.12	0.24 ± 0.41
Helicobacter	0.12 ± 0.12^a^	2.32 ± 3.17^ab^	1.71 ± 1.36^ab^	5.61 ± 3.85^b^	3.59 ± 4.78^ab^
Ruminococcaceae UCG-014	3.36 ± 1.29	2.88 ± 1.33	2.94 ± 1.87	1.48 ± 2.59	0.91 ± 1.05
Desulfovibrio	3.05 ± 1.45^a^	0.27 ± 0.27^b^	1.28 ± 1.29^ab^	0.41 ± 0.31^ab^	6.26 ± 3.55^c^
Eubacterium coprostanoligenes group	1.29 ± 1.90	1.75 ± 1.70	1.03 ± 0.51	1.68 ± 1.58	2.24 ± 2.46
Parabacteroides	0.05 ± 0.03	0.85 ± 1.14	2.56 ± 1.43	2.14 ± 2.1	1.00 ± 1.1
Allobaculum	2.33 ± 0.90^ac^	1.20 ± 0.65^ab^	0.21 ± 0.11^b^	3.23 ± 2.25^c^	0.08 ± 0.09^b^
Ruminococcaceae_uncultured	1.03 ± 0.40^ab^	0.74 ± 0.44^b^	1.65 ± 0.93^a^	0.61 ± 0.33^b^	0.38 ± 0.51^b^
Alistipes	0.16 ± 0.10	1.26 ± 1.76	0.49 ± 0.37	2.1 ± 1.8	0.14 ± 0.11
Rikenellaceae RC9 gut group	0.02 ± 0.01	1.95 ± 3.03	0.94 ± 1.00	0.90 ± 0.94	0.01 ± 0.00
Ruminiclostridium 9	0.72 ± 0.15	0.63 ± 0.12	1.61 ± 0.44	1.24 ± 0.83	0.10 ± 0.11
Lachnospiraceae_unclassified	0.23 ± 0.04^ab^	0.35 ± 0.07^a^	0.30 ± 0.12^ab^	0.18 ± 0.0.07^b^	0.15 ± 0.09^b^
Enterorhabdus	0.16 ± 0.07	0.07 ± 0.06	0.05 ± 0.03	0.08 ± 0.02	0.10 ± 0.07

A: NC group; B: 3% DSS treatment group; C: 3%DSS+p-HLP(L) group; D: 3%DSS+p-HLP(H) group; E: control+p-HLP group. There is significant difference (*P* < 0.05) if the data are labeled with different letters (a–d) in the same line.

## Data Availability

The data used to support the findings of this study are available from the corresponding authors upon request.

## Supplementary Materials

Supplementary 1 Table S1: the criteria for disease activity index (DAI) scoring.

Supplementary 2 Table S2: the evaluation criteria for histopathological scoring.

Supplementary 3 Table S3: target genes and their primer sequences.

Supplementary 4 Table S4: the glycosidic linkages of p-HLP.

Supplementary 5 Table S5: microbial diversity index.

Supplementary 6 Figure S1: effect of p-HLP on alpha diversity and microbial composition in DSS-induced colitis mice. (A–E) represent NC, DSS, DSS+p-HLP(L), DSS+p-HLP(H), and p-HLP treatment groups, respectively. (A) Rarefaction curves of the Shannon index represent species diversity, abundance, and evenness; (B) the distribution of operational taxonomic units (OTUs) among five different treatment groups is represented via a Venn diagram; (C) bacterial taxonomic profiling at the phylum level in the four groups (*n* = 4); (D) bacterial taxonomic profiling at the genus level in the four groups (*n* = 4).
